# Downregulation of SHCBP1 Inhibits Proliferation, Migration, and Invasion in Human Nasopharyngeal Carcinoma Cells

**DOI:** 10.1155/2021/8262502

**Published:** 2021-08-26

**Authors:** Tian Zhang, Xingchen He, Guodong Yu, Zhixu He

**Affiliations:** ^**1**^ Department of Pediatrics, Children's Hospital of Soochow University, Suzhou, Jiangsu 215025, China; ^**2**^ Department of ENT and HN Surgery, Affiliated Hospital of Guizhou Medical University, Guiyang, Guizhou 550002, China; ^**3**^ Department of ENT and HN Surgery, Soochow University Medical College, Suzhou, Jiangsu 215025, China

## Abstract

**Background:**

SHC SH2 domain-binding protein 1 (SHCBP1), one of the members of Src homolog and collagen homolog (Shc) family, has been reported to be overexpressed in several malignant cancers and involved in tumor progression. However, the expression of SHCBP1 in nasopharyngeal carcinoma (NPC) remains unclear, and its clinical significance remains to be further elucidated.

**Methods:**

The expression of SHCBP1 mRNA in 35 pair samples of NPC and adjacent normal tissues of NPC was detected by RT-qPCR. The expression level of SHCBP1 protein and mRNA in the selected cells was detected by western blot and RT-qPCR, respectively. The effects of SHCBP1 on NPC in vitro were observed by MTT method, colony formation assay, apoptosis assay, cell cycle assay, wound healing assay, transwell migration assay, and transwell invasion assay.

**Results:**

SHCBP1 was highly expressed in clinical tissues and NPC cell lines, and SHCBP1 knockdown significantly inhibited NPC cell proliferation. Overexpression of SHCBP1 promoted NPC cell proliferation, migration, and invasion in NPC cell lines. Silencing SHCBP1 expression can delay cell cycle and inhibit cell apoptosis.

**Conclusion:**

Our results suggest that SHCBP1 may promote proliferation and metastasis of NPC cells, which represents that SHCBP1 may act as a new indicator for predicting the prognosis of NPC and a new target for clinical treatment.

## 1. Introduction

Nasopharyngeal carcinoma (NPC) is one of the most common head and neck cancers in China. It accounts for 38.29% and 40.14% of the incidence and death of NPC in the world, respectively, with higher morbidity and mortality rates than the world average (1.2/10^5^ and 0.7/10^5^) [1]. Due to the concealed occurrence of NPC and its rapid development and high degree of malignancy, most of the patients were in the middle and advanced stages when they visited the doctor. Despite advances in diagnosis and treatment, including chemotherapy, radiation, and surgery, the 5-year relative survival rate for nasopharyngeal cancer is only 43.8% [2]. Therefore, it is urgent to elucidate the molecular mechanism involved in the progression of NPC and to identify biomarkers for early diagnosis and potential therapeutic targets.

Src homolog and collagen homolog (Shc) encode p46Shc, p52Shc, and p66Shc [3]. Each of them has a unique highly conserved structure domain PTB-CH1-SH2: a phospho-serine-binding domain (PTB), a carboxy-terminal Src homology domain (SH2), and a central proline-rich collagen-homologous region (CH1) [4, 5]. Besides, p66shc contains an amino terminal region (CH2), which plays an important role in the oxidative stress and apoptosis [6]. Multiple signaling pathways such as insulin growth factor receptor (IGFR), insulin receptor (IR), fibroblast growth factor receptor (FGFR), and epidermal growth factor receptor (EGFR) can be activated by Shc [7]. Shc plays an important part in regulating oxidative stress and various physiological functions through activation of PI3K/Akt and Ras-raf-MAPK signal pathway [3, 8, 9].

SHC SH2 domain-binding protein 1 (SHCBP1), mapped on a region of chromosome 16q11.2, is a key linker protein on the SH2 domain of the SHC protein [10]. The present study suggested that SHCBP1 may be involved in the occurrence and development of cancer [11–15]. Feng et al. [11] found that SHCBP1 was highly expressed in breast cancer and significantly correlated with the proliferation and apoptosis of the human malignant breast cancer cell line, whereas SHCBP1 knockout can restrain the proliferation of breast cancer cells. SHCBP1 was also found to be remarkably upregulated in human hepatocellular carcinoma (HCC) samples, and downregulation of SHCBP1 inhibited the proliferation and colony formation of HCC cells [12]. Dong et al. [13] found that SHCBP1 is overexpressed in GC tissues and significantly correlated with proliferation, metastatic potential, and poor prognosis. Meanwhile, several studies also confirmed that SHCBP1 is highly expressed in synovial sarcomas and may play a critical role in cell proliferation, adhesion, migration, and cell cycle progression [14, 15]. Liu et al. [16] found that EGF induces SHCBP1 into the nucleus, promotes the binding of *β*-catenin to CBP, and regulates the cell progression of non-small-cell lung cancer. In addition, studies on the mechanism of SHCBP1 in tumor growth suggested that the upregulation of SHCBP1 may be related to the activation of TGF-*β*/Smad and MEK/ERK signaling pathways [12, 15]. Together, these findings revealed that SHCBP1, as an important intracellular signaling pathway protein, plays an important role in regulating cell cycle and promoting cell migration and invasion. However, little is known about the expression and mechanism of SHCBP1 in NPC.

In the current study, we observed that SHCBP1 was significantly upregulated in NPC tissues and cell lines. SHCBP1 expression was positively associated with the cell proliferation and apoptosis. Knocking down SHCBP1 expression can promote cell apoptosis and significantly inhibit cell proliferation and invasion in vitro. Our study suggests that SHCBP1 is a tumor-promoting factor in NPC and may be a potential biomarker and therapeutic target for NPC.

## 2. Materials and Methods

### 2.1. Tissue Specimens and Cell Lines

35 pairs of NPC clinical specimens and matched peritumoral specimens were collected from The Affiliated Hospital of Guizhou Medical University and The Affiliated Cancer Hospital of Guizhou Medical University (Guiyang China) from January 2016 and December 2019. Patients did not receive chemotherapy and/or radiation prior to biopsy. Before experiments, prior consent and approval from patients and the Institutional Research Ethics Committee of Guizhou Medical University were obtained. Investigation has been conducted in accordance with the ethical standards and according to the Helsinki Declaration.

Human NPC cell lines (CNE-2Z, 5-8F) and normal nasopharyngeal cell NP69 were purchased from the Hunan Fenghui Biological Technology Co. Ltd. (Hunan China). 5-8F and NP69 were cultured in RPMI 1640 (Gibco, USA) which contained 10% fetal bovine serum (FBS, Gibco). NP69 was maintained in keratinocytes supplemented with 100 ug/ml penicillin-streptomycin (Gibco). All cells were cultured in a humidified incubator at 37°C and 5% CO_2_.

### 2.2. RT-qPCR

Total RNA was extracted. RT-qPCR was performed using a TB Green™ Premix Ex Taq™ II kit (RR820A; Takara Biotechnology Co., Ltd., Dalian, China) and detected by StepOnePlus (Applied Biosystems; Thermo Fisher Scientific, Inc.). The following conditions were used: initial denaturation at 95°C for 30 s; denaturation at 95°C for 5 s; and annealing extension of 55°C for 30 s (a total of 45 cycles). The 20 *μ*l PCR mixture was 10 *μ*l 2 × Real PCR EasyTM Mix-SYBR, 0.8 *μ*l each primer, 2 *μ*l cDNA, and 6.4 *μ*l ddH2O. At least three experiments were conducted. The data analyzed were calculated using the 2^−ΔΔCT^ method with GAPDH as an internal control [17]. The PCR primers for SHCBP1 were as follows: forward, 5′-GCTGGCGTCTCTGGAGAAAGGTTTGT-3′ and reverse, 5′-AGCAAGCCTCACCACTGCCTTCAAG-3′. The GAPDH PCR primers were as follows: forward, 5′-AGTGGTGGACCTGACCTGCCGTCTA-3′ and reverse, 5′-GGAGGAGTGGGTGTCGCTGTTGAAGT-3′.

### 2.3. Stable Cell Line Construction

Targeted shRNA sequence and negative control RNA sequence of SHCBP1 were synthesized and inserted into the lentiviral core vector expressing the GV115 reporter gene and puromycin resistance. The recombinant lentivirus was provided by Shanghai Genochemistry Co., Ltd. (Shanghai, China). The cells were infected with the corresponding lentivirus and screened with 1 g/ml puromycin for 7 days after 72 hours. The expression level of SHCBP1 in selected cells was determined by RT-qPCR and western blot.

### 2.4. MTT Assay

NPC cells were inoculated into 96-well plates at a density of 1 × 10^3^ cells/well, and the cell viability was detected by MTT (3-2,5-diphenyl tetrazolium bromide) assay (Sigma, St. Louis, USA) for 5 days. The OD was measured at the wavelength of 450 nm with a microplate reader (TEK, BioSaxony, USA).

### 2.5. Colony Formation Assay

The same number of NPC was seeded into 6-well plates at a density of 500 cells per well, respectively. The cells were then cultured in a culture dish for 2-3 weeks and cell colonies were counted (>50 cells/colony), stained with crystal violet, and photographed.

### 2.6. Apoptosis Assay

Annexin V was used to double-stain NPC cells according to the manufacturer's instructions. Cells stained with Annexin V were considered to be apoptotic. The stained cells were analyzed by flow cytometry and the data were analyzed by FACScan flow cytometry (BD Biosciences, USA).

### 2.7. Western Blotting

Cells were collected in RIPA buffer containing 100 mM Tris, 150 mM NaCl, 1 mM EDTA, 1% Triton X-100, 1% sodium deoxysulfonate, and 0.1% SDS, pH 7.4, and protease and phosphatase inhibitors were added to the mixture (Sigma-Aldrich). The protein concentration was determined by Bradford assay (Bio-Rad Laboratories, Hercules, CA, USA). The same amount of protein (25 *μ*l) was electrophoresed by 10% SDS-PAGE, transferred to a polyvinylidene fluoride (PVDF) membrane (Hybond, USA), and then probed on the membrane with the following antibodies. Antibodies against SHCBP1 (ab184467), CDK1 (ab32094), and cyclinB (ab32053) were purchased from Abcam (Cambridge, UK). The anti-*β*-actin was purchased from ABclonal (Wuhan, China). The enhanced chemiluminescence system (ECL kit, KF001, affinity) was used to detect proteins in the membrane.

### 2.8. Wound Healing Assay

NPC cells were placed in a 6-well plate at a cell density of 3 × 10^5^/ml. After 24 hours of culture, cells were infected with shCtrl, shSHCBP1, and control. The wound was scratched with a plastic straw. The cells were washed twice with phosphate buffer saline (PBS) and then incubated with serum-free RPMI 1640 medium (Gibco, USA). The cells migrated into the wounded empty space and were photographed at 0 and 24 hours after wounding. The migration rate was calculated based on the ratio of the closed wound distance to the original wound area.

### 2.9. Transwell Migration Assay

After 72 h of infection with shCtrl, shSHCBP1, and control, cells were collected and resuspended in serum-free medium. Then cells were added to the upper chamber at a density 5 × 10^5^ cells/ml (200 *μ*l per chamber), and 600 *μ*l of medium containing 10% fetal bovine serum was added to the lower chamber. Cells migrated for 24 h in a CO_2_ incubator at 37°C. Then the migrating cells on the bottom surface were fixed with methanol and stained with 0.1% crystal violet, and 5 microscope fields were randomly selected for counting in each well.

### 2.10. Transwell Invasion Assay

An 8.0 m well transwell insert (Millipore, Billerica, MA, USA) is precoated with 100 *μ*l 200 *μ*g/ml Matrigel (BD Biosciences, Franklin Lakes, NJ, USA) and put it in a 24-well plate at room temperature for 60 minutes. After 72 h of infection with shCtrl, shSHCBP1, and control, the cells were collected and resuspended in serum-free medium. 5 random field invading cells were counted in each chamber, and pictures were taken under a light microscope at 200 times.

### 2.11. Statistical Analysis

All experiments were conducted independently at least three times. Statistical analysis was performed using Social Science Statistical Software Package (SPSS) 20.0 software (SPSS Inc., Chicago, IL) and Prism 5.0 software (GraphPad software, La Jolla, CA). Student's *t*-test was used for comparison between the two groups. One-way ANOVA was used to compare data consisting of more than two groups. Pearson *χ*^2^ test and Log-rank test were used to evaluate the statistical differences. The data displayed is expressed as mean ± standard deviation (SD). *p* < 0.05 was considered statistically significant.

## 3. Results

### 3.1. Increased Expression of SHCBP1 in NPC Tissues and Cell Lines

To determine the expression pattern of SHCBP1 in NPC tissues, we compared the relative mRNA levels of SHCBP1 in 35 pairs of matched NPC tissue samples using RT-qPCR. Compared with adjacent nontumor tissues, SHCBP1 in tumor tissues was significantly upregulated (Figure 1(a)). In addition, we found that SHCBP1 expression was higher in CNE-2Z and 5-8F cells compared with NP 69 cells (Figure 1(b)). The results showed that, in NPC tissues and cell lines, the relative expression of SHCBP1 mRNA was significantly increased. For further functional experimentation, we selected 5-8F cells with a lower expression of SHCBP1 for the experiment. 5-8F cell lines were selected to construct knockdown models.

### 3.2. SHCBP1 Promoted Proliferation and Colony Formation of NPC Cells

To explore the effect of downregulation of SHCBP1 gene on the proliferation of NPC cells, shRNA was used to downregulate the expression of endogenous SHCBP1 gene in 5-8F cell lines. shRNA was transfected into NPC cells and RT-qPCR was used to evaluate the efficiency of interference. The shRNA interference significantly reduced the SHCBP1 mRNA expression level of 5-8F cells compared with the knockdown control group (shCtrl) (Figure 2(a)). Downregulation of SHCBP1 significantly inhibited the growth of 5-8F cells compared with shCtrl (Figure 2(b)). shCtrl and shSHCBP1 were used to assay cellular proliferation. MTT assay and Celigo assay inhibited SHCBP1 expression for 5 days and significantly inhibited 5-8F cell proliferation (Figures 2(c)-2(e)). Therefore, the above data suggested that knocking down SHCBP1 can inhibit the proliferation of NPC cells.

In order to explore the effect of SHCBP1 on the colony formation in NPC cell, 5-8F cells treated with SHCBP1-shRNA or control-shRNA lentivirus were allowed to grow for 14 days to form colonies. Compared with the control group (shctrl), the number of cell colonies in the knockdown group (shSHCBP1) was reduced, suggesting that SHCBP1 was largely correlated with the clonal formation ability of NPC cells (Figures 2(f) and 2(g)). The above data implied that SHCBP1 may play a key role in colony formation of NPC cells.

### 3.3. SHCBP1 Suppressed Apoptosis in NPC Cells

Using Annexin V-APC stained with FACS in 5-8F cells after lentivirus infection, the effect of SHCBP1 on cell apoptosis was explored (Figure 3(a)). As shown in Figure 3(b), the apoptotic rate of SHCBP1-shRNA lentivirus-infected cells was significantly higher than that of shctrl lentivirus-infected cells, and the apoptotic rate was significantly different between shctrl and shSHCBP1 (*p* < 0.05). Flow cytometry analysis showed that inhibition of SCHBP1 expression can significantly induce apoptosis of NPC cells.

### 3.4. SHCBP1 Was Required in Migration and Invasion of NPC Cells

To investigate the role of SHCBP1 in sinus cell migration, the effect of SHCBP1 knockout on migration ability was examined in the wound healing assay. Compared with shCtrl, the migration distance of shSHCBP1 (Figure 4(a)) cells was significantly reduced. In the invasion and metastasis assay, we evaluated the invasion and migration ability of 5-8F cells treated with transwell. Compared with shCtrl cells, the number of cells invaded and migrated by shSHCBP1 cells was significantly reduced (Figure 4(b)). These data suggest that reduced SHCBP1 expression inhibits the invasion and metastasis of NPC cells.

### 3.5. SHCBP1 Promoted Cell Cycle with Increased Expressions of CDK1 and Cyclin B

In order to further explore the molecular mechanism of SHCBP1 regulating NPC cell cycle, we detected the expression levels of CDK1 and cyclin B, key proteins in cell cycle regulation, by western blot (Figure 5(a)). As Figure 5(b) showed, it was found that the expressions of CDK1 and cyclinB were lower in the knockdown group (shSHCBP1) than in the knockdown control group (shctrl) (*p* < 0.05). The results indicated that SHCBP1 may stimulate cell cycle progression via upregulation of CDK1 and cyclin B.

## 4. Discussion

Although the mortality rate of NPC has decreased with the improvement of diagnosis and treatment, NPC is still one of the most deadly head and neck malignancies in adults, mainly because the specific molecular pathogenesis has not been fully elucidated and due to the lack of targeted therapy [18, 19]. In recent years, the upregulation of SHCBP1 has been shown to be associated with malignant transformation in many types of tumors [11–15]. In this work, we found that SHCBP1 was upregulated in NPC tissues compared with that of adjacent nontumor tissues. Furthermore, we found that the expression of SHCBP1 was higher in CNE-2Z and 5-8F cells compared with that of NP 69 cells. These results are consistent with previous studies that have shown that elevated SHCBP1 expression is detected in a variety of cancers and may have implications for early diagnosis [11–15]. Therefore, SHCBP1 can be used as a potential therapeutic target for NPC and may be helpful for the diagnosis and prognosis of NPC. To the best of our knowledge, this is the first time that the role of SHCBP1 in NPC has been revealed. The relationship between SHCBP1 expression and the clinical characteristics of NPC is worth further study.

In order to explore whether SHCBP1 plays a role in the proliferation and colony formation of NPC cells, we used shRNA to knock down SHCBP1 in the endogenous 5-8F cell line. Then MTT assay and Celigo assay were used to evaluate the effect of interfering with SHCBP1 expression on the proliferation and colony formation of NPC cells. Furthermore, wound healing assay, flow cytometry, and transwell assay were used to evaluate the effect of knockdown of SHCBP1 on migration and invasion of NPC cells. We found that reducing SHCBP1 expression significantly reduced the migration and invasion of NPC cells. Therefore, knockout of SHCBP1 might prevent NPC by inhibiting the metastasis and invasion of NPC cells.

Defects in apoptosis mechanisms play important roles in tumor pathogenesis, allowing neoplastic cells to survive over intended lifespans [20]. Cyclin B, the key cell cycle regulating protein, could accumulate in the S and G2 phases to form an inactive mitosis-promoting factor (MPF) with CDK1 during the normal cell cycle stages [21]. In this study, we found that silencing SHCBP1 can significantly inhibit the expression of CDK1 and cyclin B in NPC cells. These results reveal that the mechanism of SHCBP1-mediated proliferation and apoptosis may be related to the alternations of the expression of cyclin B and CDK1.

The molecular mechanism that underlies the development of NPC is not fully understood. It is traditionally believed that the occurrence and development of NPC are related to Epstein–Barr virus infection environment and diet, local chronic inflammation, and so on. Recently, the molecular targeted therapy of vascular endothelial growth factor receptor (VEGFR), epidermal growth factor receptor (EGFR) family, and PI3K/Akt/mTOR emerged, whereas the side effect is much; curative effect is still not ideal. Previous research suggests that PI3K/Akt TGF-*β*/Smad, NF-*κ*B signaling pathways, and EGFR mutations are involved in promoting the growth, proliferation, metastasis, cell cycle, and apoptosis of NPC cells [22–24]. Therefore, it is urgent to find new therapeutic targets. For the first time we reported the association between SHCBP1 and NPC. At present, our laboratory is further exploring the possible molecular mechanism of SHCBP1 in the proliferation and invasion of NPC cells.

## 5. Conclusion

SHCBP1 is significantly upregulated in clinical NPC cell lines and tumor samples. Reducing SHCBP1 expression can inhibit cell proliferation and metastasis, induce apoptosis, and suppress cell cycle in NPC cell lines, suggesting that SHCBP1 may be linked to NPC progression and serve as a potential biomarker and therapeutic target for NPC.

## Figures and Tables

**Figure 1:** High expression of SHCBP1 in NPC tissues and cell lines. (a) RT-qPCR analysis of SHCBP1 in NPC clinical specimens and the paired normal nasopharyngeal tissues (^*∗*^*p* < 0.05). (b) RT-qPCR analysis of SHCBP1 mRNA in NPC cell lines (5-8F and CNE-2Z) and in normal nasopharyngeal cells (NP69). ^*∗∗*^*p* < 0.01 vs. NP69 group. Data are presented as mean ± SD.

**Figure 2:** SHCBP1 knockdown inhibited cellular proliferation and colony formation of NPC cells. (a) SHCBP1 mRNA levels were significantly lower in the knockdown group (shSHCBP1) than in the control group (shCtrl) after lentivirus infection (^*∗∗*^*p* < 0.01). (b) 5-8F cells transfected with negative control lentivirus (shCtrl) and SHCBP1 knockdown lentivirus (shSHCBP1) were transfected and knocked out by lentivirus (SHSHCBP1) and photographed under x100. (c, d) MTT was used to detect the cell activity of shCtrl and shSHCBP1. (e) Celigo detected the number of cells in shCtrl and shSHCBP1 at each time point. (f) Colony formation assays revealed that shSHCBP1 had a better effect on the proliferation of 5-8F cells than shCtrl. (g) The number of colonies in F was analyzed (^*∗∗*^*p* < 0.01). SHCBP1, SHC SH2 domain-binding protein 1; NPC, nasopharyngeal carcinoma; shSHCBP1, SHCBP1-shRNA; shCtrl, negative control-shRNA.

**Figure 3:** SHCBP1 suppression induced apoptosis in NPC cells. (a) Cells stained with Annexin V were apoptotic cells. (b) The apoptotic index was defined as the percentage of apoptotic cells. Values are mean ± SD of 3 independent experiments (^*∗∗*^*p* < 0.01). SHCBP1, SHC SH2 domain-binding protein 1; NPC, nasopharyngeal carcinoma; shSHCBP1, SHCBP1-shRNA; shCtrl, negative control-shRN.

**Figure 4:** SHCBP1 knockdown inhibited migration and invasion of NPC cells. (a) In the wound healing test, at 0 hours and 24 hours, representative micrographs of shSHCBP1 cell movement compared with untreated cells and vehicle control cells. (b, c) Transwell assays examined cell migration (b) and invasion (c) after SHCBP1 knockdown. SHCBP1, SHC SH2 domain-binding protein 1; NPC, nasopharyngeal carcinoma; shSHCBP1, SHCBP1-shRNA; shCtrl, negative control-shRNA.

**Figure 5:** SHCBP1 influenced cell cycle progression of NPC cells. (a, b) The levels of CDK1 and cyclin B were detected in control (1), shCtrl (2), and shSHCBP1 (3) cells by western blot analysis. *β*-Actin was used as the loading control. Values are mean ± SD of 3 independent experiments; ^*∗*^*p* < 0.05; ^*∗∗*^*p* < 0.01. SHCBP1, SHC SH2 domain-binding protein 1; NPC, nasopharyngeal carcinoma; shSHCBP1, SHCBP1-shRNA; shCtrl, negative control-shRNA.

## Data Availability

The data used and/or analyzed during the current study are available from the corresponding author upon request.
